# Expression of SARS-CoV-2 Spike Protein Receptor Binding Domain on Recombinant *B. subtilis* on Spore Surface: A Potential COVID-19 Oral Vaccine Candidate

This article has been retracted.

**DOI:** 10.3390/vaccines10010002

**Published:** 2021-12-21

**Authors:** Johnny Chun-Chau Sung, Ying Liu, Kam-Chau Wu, Man-Chung Choi, Chloe Ho-Yi Ma, Jayman Lin, Emily Isabel Cheng He, David Yiu-Ming Leung, Eric Tung-Po Sze, Yusuf Khwaja Hamied, Dominic Man-Kit Lam, Keith Wai-Yeung Kwong

**Affiliations:** 1 Research Department, DreamTec Cytokines Limited, Hong Kong, China; johnnysung@dreamtec.hk (J.C.-C.S.); liuying@dreamtec.hk (Y.L.); kcwu@dreamtec.hk (K.-C.W.); jerrychoi@dreamtec.hk (M.-C.C.); Chloema@dreamtec.hk (C.H.-Y.M.); jaymanlin@dreamtec.hk (J.L.); info@dreamtec.hk (E.I.C.H.); 2 Oristry BioTech (HK) Limited, Hong Kong, China; 3 Meserna Therapeutic (HK) Limited, Hong Kong, China; 4 L&L Immunotherapy Company Limited, Hong Kong, China; dlam@worldeye.org; 5 Zentrogene Bioscience Laboratory Limited, Hong Kong, China; davidleung@hpm.com.hk; 6 Health Plus Laboratory Limited, Hong Kong, China; 7 School of Science and Technology, Hong Kong Metropolitan University, Hong Kong, China; esze@hkmu.edu.hk; 8 Cipla Limited, Mumbai 400013, India; ykh@cipla.com; 9 Torsten Wiesel International Research Institute, Sichuan University, Chengdu 610017, China

**Keywords:** SARS-CoV-2, COVID-19, oral vaccine, *Bacillus subtilis*, spike protein, sporulation

## Abstract

Various types of vaccines, such as mRNA, adenovirus, and inactivated virus by injection, have been developed to prevent SARS-CoV-2 infection. Although some of them have already been approved under the COVID-19 pandemic, various drawbacks, including severe side effects and the requirement for sub-zero temperature storage, may hinder their applications. *Bacillus subtilis* (*B. subtilis*) is generally recognized as a safe and endotoxin-free Gram-positive bacterium that has been extensively employed as a host for the expression of recombinant proteins. Its dormant spores are extraordinarily resistant to the harsh environment in the gastrointestinal tract. This feature makes it an ideal carrier for oral administration in resisting this acidic environment and for release in the intestine. In this study, an engineered *B. subtilis* spore expressing the SARS-CoV-2 spike protein receptor binding domain (sRBD) on the spore surface was developed. In a pilot test, no adverse health event was observed in either mice or healthy human volunteers after three oral courses of *B. subtilis* spores. Significant increases in neutralizing antibody against sRBD, in both mice and human volunteers, after oral administration were also found. These findings may enable the further clinical developments of *B. subtilis* spores as an oral vaccine candidate against COVID-19 in the future.

## 1. Introduction

*Bacillus subtilis* (*B. subtilis*) is a Gram-positive and endophytic sporoforming bacterium, many strains of which have been proven to possess probiotic properties [1]. Under starvation, dormant spores of *B. subtilis* are formed, which can resist the harsh environmental conditions in the gastrointestinal tract [2]. Hence, this enables *B. subtilis* to be colonized in the intestinal tract of the human body [3]. Probiotic strains of *B. subtilis* are involved in the maintenance of the intestine’s microecological balance [4], and can stimulate the release of secreted immunoglobulin [5], which is conducive to the local immunity of intestinal mucosa [6] and enhances the immunity of the human body [7]. Due to its characteristics in regulating humoral and cellular immunity, *B. subtilis* has become an ideal vaccine carrier for the mucosal immunization vaccine [8]. Together with its GRAS (generally considered as safe) property (in certain strains) and easy genetic manipulationproperties, this organism can serve as an ideal platform for the heterologous expression of bioactive substances in the intestinal tract [9]. *B. subtilis* has been used as an adjuvant in chickens treated with inactivated avian influenza virus H9N2 [10]. The use of recombinant *B. subtilis* has become an economical and practical solution, as it can be mass-produced, due to its easy cultivation [11] and safety [12]. It has been applied in industry [13], agriculture [14], medicine [15], health and food [16] and other fields [17,18].

Experimental reports have supported that there are no significant adverse effects caused by probiotic strains of *B. subtilis* in acute toxicity tests [19,20] or in organs [21], such as the heart and liver, indicating that *B. subtilis* is safe and non-toxic to mammals [22]. It has also been reported that specific oral serum IgG and intestinal mucosal SIgA, in mice, can be induced by the administration of recombinant *B. subtilis* spores [23].

Coronavirus disease (COVID-19) is a serious global pandemic, with an estimated 226.61 million confirmed cases of infection and 4.66 million deaths as of September 2021. Due to the lack of effective drug treatments, the development and use of COVID-19 vaccines have become an important strategy for controlling the COVID-19 outbreak [24]. Coronavirus is a class of enveloped viruses with positive-sense single-stranded RNA [25]. The receptor-binding domain on the spike protein expressed on the envelop is the major target for neutralization by antibodies [26]. In March 2020, COVID-19 vaccines, based on an adenovirus vector, in China, [27] and an mRNA technology platform in the United States [28], were the earliest batches of candidates to enter clinical trials, followed by a DNA-type vaccine [29] and an inactivated vaccine [30]. At present, 60 vaccine candidates, based on six different major technical routes—namely, inactivated virus vaccines, nucleic acid vaccines (including DNA and mRNA vaccines), vector vaccines, protein subunit vaccines, live attenuated vaccines and virus-like particle vaccines—have been approved for clinical trials [31,32]. Some vaccines have been granted conditional marketing authorization [33] or emergency use authorization [34].

The safety of COVID-19 vaccines is under scrutiny [35,36]. In general, inactivated and protein subunit-type vaccines do not cause viral infection. Live attenuated-type vaccines, on the other hand, need to be reproduced in vivo, which carries the risk of virulence atavism or transmission [37]. Therefore, vaccines made of inactivated virus and protein subunit are generally safer than live attenuated-type vaccines. Protein subunit-type vaccines are more accurate in composition and slightly safer than inactivated virus vaccines. DNA-type vaccines, which belong to nucleic acid vaccines, have the risk of oncogene activation, tumor suppressor gene inactivation, and chromosome instability. These may be caused by the integration of foreign DNA into the host genome after entering the body [29]. The synthetic materials and encapsulated liposomes used in the synthesis of mRNA vaccines may be cytotoxic and cause apoptosis of the surrounding host cells. Non-replicating adenovirus vector vaccines are relatively safe as they cannot replicate by themselves. However, due to the wide range of adenovirus infections and lack of targeting, adenovirus vectors may infect other normal tissue cells, resulting in adverse effects [38]. In addition, attention needs to be paid to the antibody-dependent enhancement (ADE) effect when developing COVID-19 vaccines, especially in inactivated vaccines. Although there is still no COVID-19 vaccine-related ADE reported, similar phenomena have been observed in MERS [39] and SARS vaccine candidates [40]. Based on the results of the phase I/II clinical trials of the current vaccine candidates, it is noteworthy that a very rare brand-new type of adverse effect, thrombocytopenia syndrome [41], has been observed. This involves abnormal and severe coagulation events with low platelet counts, which occur following the administration of the viral vector vaccine Vaxzevria. The biological mechanism of thrombocytopenia syndrome is still under investigation. At this stage, the “platform-specific” mechanisms associated with adenovirus vector vaccines are uncertain but cannot be ruled out. Another concern is the storage conditions of vaccines. Due to the instability and easy degradation of mRNA, mRNA vaccines have high requirements for storage conditions [42]. An mRNA-type vaccine jointly developed by the United States and Germany needs to be stored at −70 °C [43]. After they are thawed, the vaccine vials can only be stored for 5 days in cold storage (2~8 °C). Another mRNA vaccine was only stable for 30 days at 2 to 8 °C and needed to be stored at −20 °C.

In addition to the safety and storage constraints of different types of vaccines, a sufficient supply of vaccines to different parts of the world is also a major challenge to the pandemic, as billions of individuals from poorer countries do not have access to COVID-19 vaccines, which could raise the risk of the development of variants of the virus [44]. The prices of COVID-19 vaccines range from USD 5 to 62, which may not be affordable to individuals in many developing counties, prohibiting them from completing a two-dose vaccination schedule.

Twenty years ago, our group began to investigate the possibilities of employing edible plants, yeast and lactobacillus as oral vaccine candidates [45,46,47,48,49,50,51]. There is currently no commercially available vaccine made of a specific expression vector in *B. subtilis,* nor an orally administrated-type vaccine for COVID-19 prophylaxis. The use of *B. subtilis* as a vector is better than adenovirus, as *B. subtilis* is relatively safe. Additionally, it would not cause any blood coagulation event as the bacterial vector would not enter the bloodstream. *B. subtilis* vaccines also have a lower production cost. Therefore, we believe that oral *B. subtilis* vaccines will make a significant contribution to the prevention and treatment of COVID-19 in the future. There is currently no commercially available vaccine made of a specific expression vector in *B. subtilis* or an orally administrated-type vaccine for COVID-19 prophylaxis. The use of *B. subtilis* as a vector is better than an adenovirus, as *B. subtilis* is relatively safe. Additionally, it would not cause any blood coagulation event, as the bacterial vector would not enter into the bloodstream. *B. subtilis* vaccines also have a lower production cost. Freeze-dried *B. subtilis* spores in capsules are stable for long-term storage under ambient conditions [52]. Therefore, we believe that oral *B. subtilis* vaccines could be a potential candidate for the treatment of COVID-19. The advantages of using genetically modified *B. subtilis* spores as the vector of vaccines can make a significant contribution to the prevention and treatment of diseases in the future.

In this study, we proved that the sRBD of SARS-CoV-2 can be expressed on the genetically engineered *B. subtilis* spore surface, which can successfully induce neutralizing antibody against sRBD in mice. A human pilot study was conducted, wherein daily 1 × 10^9^ recombinant oral administration of this *B. subtilis* spore did not cause any significant adverse health effects and could successfully induce significant neutralizing antibodies in human volunteers who had not been vaccinated. The experiment proved that the engineered *B. subtilis* can be a potential oral vaccine for COVID-19, where the results from the study can be used for the design of further clinical trials. Furthermore, to the best of our knowledge, this is the first successful example of a *B. subtilis* oral vaccine being tested on humans.

## 2. Materials and Methods

### 2.1. Construction of Recombinant B. subtilis Spores

Unless otherwise specified, all chemicals were purchased from Sigma-Aldrich (St. Louis, MO, USA). CDS of sRBD from SARS-CoV-2 (Wuhan-Hu-1, Clade 19, a.a. 319–541, UniProt ID: P0DTC2) [53] was codon-optimized for *B. subtilis* and synthesized by the GeneArt Gene synthesis service (Thermo Fisher Scientific, Waltham, MA, USA). A linker peptide of -GGGEAAAKGGG- was used to fuse the sRBD with the CDS of *CotA*, *CotB*, or *CotC* from the C-terminal and cloned into pHT01 (MoBiTec, Gottingen, Germany). The cloned plasmids were transformed into *B. subtilis* strain WB800N (MoBiTec, Gottingen, Germany) according to the manufacturer’s instructions.

To generate the spores expressing the recombinant proteins, transformed *B. subtilis* was inoculated and fermented with 2 × LB supplied with 0.5% glucose in a bioreactor. The cells were harvested when OD600 reached 8 and centrifuged at 4200× *g* for 10 min and washed once with PBS. The cell pellet was then resuspended in Difco’s sporulation medium [54] supplied with 1 mM IPTG, and shaken at 250 rpm at 37 °C for 48 h to produce recombinant spores. After sporulation, the spores were incubated with 15 µg/mL lysozyme in PBS to lyse the vegetative *B. subtilis* cells. The resulting spores were centrifuged at 4200× *g* for 10 min and washed five times with PBS before lyophilizing.

### 2.2. Characterization of Recombinant B. subtilis Spores

The counting of spores was performed in triplicate in a hemocytometer and the average was taken. To extract the coat proteins for Western blot analysis, the freeze-dried spores were decoated with SD solution (1% SDS, 50 mM DTT) at 70 °C for 1 h with occasional mixing [55]. The decoated spores were then centrifuged at 14,800× *g* for 10 min. The resulted supernatant was added with 4× SDS-PAGE loading buffer and subjected to Western blot analysis with rabbit-anti-SARS-CoV-2 Spike RBD antibody (Sino Biological Beijing, China, cat. no. 40592-T62, 1:5000 dilution). Then, 100 ng of sRBD standard was loaded as a positive control (Sino Biological, Beijing, China, cat. no. 40592-V08B).

For immuno-staining, the spores were resuspended in PBS and blocked with 5% normal goat serum in PBS for 1 h at room temperature. The spores were then stained with rabbit-anti-SARS-CoV-2 Spike RBD antibody (1:500 dilution) followed by AF488 conjugated donkey–anti-rabbit IgG (H + L) (Invitrogen, cat. no. R37118, 1:1000) and subjected to fluorescent microscopy or FACS analysis.

### 2.3. Cytokine Profiling of Dendritic Cells

Monocytes were plated at 2 × 10^6^ per ml in a 24-well plate and allowed to adhere for 45 min, at 37 °C and 5% CO_2_. Non-adherent cells were removed by washing the wells thrice with a gentle stream of medium. Monocytes were then cultured in the presence of granulocyte macrophage colony-stimulating factor (50 ng/mL) and IL-4 (40 ng/mL) at 37 °C under 5% CO_2_. On day 3, 50% of the medium was replaced with fresh medium and cytokines. Dendritic cells (DCs) were then harvested on day 6 and washed. The cells were then treated with peptidoglycan from B. subtilis (2.5 μg/mL), recombinant spores, or PBS control for 48 h. The supernatants from DCs cultures were collected and stored at −80 °C until assayed for cytokines. The levels of IL-1β, IL-6, IL-10, and TNF-α were measured in duplicate with Bio-plex human cytokine/chemokine multiplex assay with a Bio-plex 200 System (Bio-Rad, Hercules, CA, USA).

### 2.4. Immunization of Mice

All animal experiments were conducted according to relevant national and international guidelines. The animal protocols used have been reviewed and approved by the Animal Ethics Committee of The Chinese University of Hong Kong. Furthermore, 8-week-old BALB/c mice were orally administered 1 *×* 10^9^ spores/kg mice with a stainless-steel round-tip gavage cannula at days 1–3, 14–16 and 28–30. The mice were monitored on a daily basis for clinical changes, including body weight, hair loss, body temperatures, eating habits and diarrhea.

Mice were bled under general anesthesia at days 0, 8, 22, and 38. To determine the titers of serum antibodies, ELISA plates were coated with sRBD standard (0.1 ng/well). Serially diluted sera in 1% BSA in PBS were added to wells of the coated plate and incubated for 1 h at room temperature. Goat anti-mouse IgG conjugated with alkaline phosphatase (Southern Biotechnology, Birmingham, AL, USA) served as secondary antibodies. The antibody titer was defined as the highest serum dilution showing an absorbance of 0.1 or greater of that of normal sera. A response was considered positive by ELISA if the titer of reactivity increased from the undetectable pretreatment to at least 1:40 after vaccination, or from the detectable pretreatment by 8-fold.

### 2.5. Immunization of Human

All human experiments were conducted according to relevant national and international guidelines. Written consent was obtained from all volunteers. The protocols used were reviewed and approved by Doctors Think Tank Academy Ethic Committees and the Research Ethics Committee of the Hong Kong Metropolitan University. Volunteers were orally administered 5 × 10^7^ spores/kg person of recombinant *B. subtilis spores* mixed with sodium alginate in enteric coated capsules at days 1, 14 and 28. Furthermore, 5-mL blood samples were drawn at days 0, 27 and 42, and the serum samples were stored at −80 °C until assay. The titer of neutralizing antibodies was determined with a CLIA-based assay MAGLUMI SARS-CoV-2 Neutralizing Antibody detection kit (Snibe Dianostic Shenzhen, China).

The neutralizing capabilities of immunized volunteers towards SARS-CoV-2 were assessed with a lentiviral pseudovirus neutralization assay. Pseudoviruses with the SARS-CoV-2 Spike protein and a GFP reporter gene were produced in HEK293T cells according to the manufacturer’s instructions (InvivoGen, Hong Kong, China, cat. no. PLV-SPIKE). Approximately 1 × 10^5^ infectious units of pseudoviruses were pre-incubated with serial diluted serum from volunteers for 1 h at 37 °C. Human lung carcinoma cell line A549 expressing ACE2 and TMPRSS2 (InvivoGen, cat. no. A549-HACE2TPSA) was plated in a 96-well plate at a density of 1 × 10^5^/well and incubated with pre-incubated pseudoviruses. At 2 days post-infection, the plates were analyzed with a fluorescent plate reader with the GFP filter set. A non-linear regression was performed for the response curve of the infection percentage to the dilution of sera. The serum titer that resulted in 50% infection is reported as the EC_50_.

### 2.6. Statistical Analysis

Data are expressed as the mean ± SEM, and statistical significance was determined by a student’s t-test, and one-way or two-way ANOVAs with Tukey’s post hoc test in GraphPad Prism 7.1 (La Jolla, CA, USA). Data were considered significantly different when the *p*-value was less than 0.05.

## 3. Results

### 3.1. Establishment of the Surface-Displaying Antigen Model of Bacillus subtilis Spore

To develop recombinant *B. subtilis* spores displaying antigens from SARS-CoV-2, we designed an expression cassette under the control of an inducible promoter _p_grac in a shuttle vector pHT01. To maximize the production of neutralizing antibodies against SARS-CoV-2, we decided to express sRBD from SARS-CoV-2 [56,57] linked to different coat proteins from *B. subtilis* for the surface display of sRBD [58]. Three different coat proteins, CotA, CotB, and CotC, were linked with sRBD and inserted into the pHT01 vector (Figure 1A) followed by transformation into *B. subtilis*. The schematic of spore production is shown in Figure 1B and described in detail in the Materials and Methods section. Western blot analysis of the recombinant spores showed that the expression of the CotC-linked sRBD was much higher, while the CotA or CotB-linked sRBD was not detectable (Figure 1C). This is possibly due to the selection of coat proteins, the linker region and the fusion protein [59,60,61]. Subsequently, the expression of CotC-sRBD was tested in a time-course experiment for the time of sporulation. The *B. subtilis* transformed with pHT-01-DT-C-sRBD was subjected to sporulation in Difco Sporulation Medium (DSM) and to 1mM IPTG for protein expression. Spores were then harvested for Western blot analysis. Starting from 4 h of induction, the expression of CotC-sRBD was detectable and was found to peak at 24 h (Figure 1D).

To validate the display of the sRBD protein on the surface of the recombinant spores, an immunofluorescent staining of the recombinant spores was performed. *B. subtilis* transformed with the pHT01 empty vector; constructs with CotA-, CotB- or CotC-linked sRBD were induced into spores. The spores were then stained with anti-sRBD primary antibody followed by Alexa Flour 488-conjugated secondary antibody and subjected to fluorescent microscopy. Consistent with the Western blot analysis, only the spores expressing CotC-linked sRBD were immunoreactive, but not the native, CotA- or CotB-linked sRBD spores (Figure 2A). The spores expressing CotC-linked sRBD were also analyzed with flow cytometry and showed the same result (Figure 2B). These results confirmed that the CotC-linked sRBD proteins were displayed on the surface of the recombinant spores.

### 3.2. Immunoreactivity of B. subtilis Spores in Cells and Mice

To assay the immunoreactivity of *B. subtilis* spores, different models were studied. As proteins on the *B. subtilis* may serve as immunogenic adjuvants that can promote cytokine and chemokine secretions in dendritic cells (DCs) [62,63], we first tested if the peptidoglycan from *B. subtilis* (PGN-BS) can provoke cytokine secretion. Purified DCs were cultured and incubated with PGN-BS or PBS as a control for 48 h before harvesting the culture medium for cytokine profiling. The results showed that incubation with PGN-BS significantly increased the proinflammatory factors TNF-α, IL-1β, IL-6, and IL-10 compared to the control group (Figure 3A). To test the possible adjuvant effect of *B. subtilis*, DCs with a potent Toll-like receptor agonist were co-treated with polyinosinic–polycytidylic acid high-molecular weight [poly(I:C) HMW], together with PGN-BS. While the incubation with poly(I:C) HMW alone could promote the secretion of TNF-α, IL-1β, IL-6, and IL-10, co-treatment with PGN-BS significantly boosted the levels of proinflammatory factors (Figure 3B). To further confirm the adjuvant capability of *B. subtilis* spores, we also treated the DCs with the recombinant *B. subtilis* spores co-treated with [poly(I:C) HMW]. Similar to treatment with PGN-BS, the treatment of recombinant spores could provoke the secretion of TNF-α, IL-1β, IL-6, and IL-10 (Figure 3C). This suggested that the *B. subtilis* can promote the immune response and has an immune-adjuvant effect.

A mice pilot test was then conducted to test the specific immunoreactivity of the recombinant *B. subtilis* spores in mice. Eight-week-old BALB/c mice (*n* = 4) were orally administrated with *B. subtilis* spores expressing CotC-sRBD for three courses (days 1–3, days 14–16 and days 28–30), and blood samples were drawn at days 0, 8, 22, and 38 (Figure 4A). The sera of the blood samples were then analyzed by enzyme-linked immunosorbent assay (ELISA) to determine the levels of antibodies against sRBD. No adverse effect, such as fatality, fever, weight loss or diarrhea, was observed in mice treated with recombinant *B. subtilis* spores. ELISA results showed a significant increase in IgG against sRBD over time starting from day 22 (F = 20.22, *p* < 0.001, two-way ANOVA) (Figure 4B). IgA against sRBD was also detectable in both serum and intestinal lavage (unpublished data) after the three courses of oral administration. The data suggested that recombinant spores can promote the production of antibodies against sRBD in mice, which can be used as a novel vaccination strategy.

### 3.3. Protection Effect of Recombinant B. subtilis Spores against SARS-CoV-2

As *B. subtilis* WB800N is considered as a GRAS food ingredient [64], six healthy, unvaccinated individuals, aged between 48 and 72 years old, were recruited. The volunteers took three courses of 5 × 10^7^ spores/kg person *B. subtilis* spores via oral administration, and their serum samples were collected as indicated in Figure 5A. The serum samples were then subjected to a chemiluminescence light immunoassay (CLIA) to measure the titer of antibodies targeting the RBD of SARS-CoV-2. The CLIA results showed that, after the second dose of oral vaccination, there was an observable increase in the neutralizing antibodies at day 27. After the third dose of oral vaccination, there was a significant increase in neutralizing antibody in the serum (F = 24.96, *p* < 0.001, two-way ANOVA) (Figure 5B). The ability to neutralize against SARS-CoV-2 was tested by an in-vitro pseudovirus neutralization assay. Lentivirus, carrying a GFP gene, was pseudotyped with the spike protein from a wild-type or D614G variant of SARS-CoV-2. The pseudoviruses were then pre-incubated with serially diluted serum samples from orally vaccinated volunteers before being added to A549 lung carcinoma cells expressing human ACE2 and human TMPRSS2. The percentage of infection rate was measured with a fluorescent microscope by counting GFP-positive cells. Representative plots of the neutralization assay with wild type and D614G are shown in Figure 5C,D, respectively. Coherent with the antibody titer result, 27 days post-vaccination, undiluted sera were able to neutralize and prevent the infection of the pseudovirus, and to a much higher extent at 42 days post-vaccination both for wild type (F = 18.91, *p* < 0.001, two-way ANOVA) and D614G (F = 31.83, *p* < 0.001, two-way ANOVA) pseudoviruses (Figure 5C,D). A regression model was applied to the neutralization assay result to find the EC50 value of the reciprocal of the serum dilution (Figure 5E,F). The data showed that after three courses of oral vaccination, the sera from vaccinated volunteers could neutralize and block the infection of the SARS-CoV-2 pseudovirus in vitro.

## 4. Discussion

As the pandemic caused by the COVID-19 virus has spread globally [65] for nearly two years, the prevalence rates continue to rise [66]. Vaccinations for COVID-19 are currently the most effective means of controlling the spread of the disease [67], with more than 200 vaccines in different forms currently in development around the world [68]. Although some of these vaccines have been quickly approved for marketing through the EUA pathway [69], the stability, safety and efficacy of these vaccines are still being explored. Therefore, the development of a safe, economic, effective and stable vaccine will be a potential solution.

Drug manufacturing using genetically modified organisms, such as *Escherichia coli*, has been used for a long time, where the oral administration of some genetically modified gut microbiomes has become an emerging technique in therapeutic applications. For example, an engineered *Escherichia coli* strain, SYNB1020, was shown to have no adverse events and a dose-dependent effect in producing arginine [70]. The use of orally administered genetically engineered bacterial vaccines is an attractive strategy for generating a stronger immune response compared to vaccines using the inactivated virus. Extra-gastrointestinal mucosal stimulation has been used to evaluate the optimal immunity against different pathogens. Mucosal promotion strategies are usually obtained by a live replication delivery system or by combining soluble antigens with a potent mucosal adjuvant, such as cholera toxin (CT) [71] or *Escherichia coli* [72], heat-intolerant enterotoxin or their derivatives. However, due to the toxicity of these adjuvant toxins, they are not suitable for human use, and the use of soluble antigens alone tends to establish immune tolerance rather than immunity [73].

*B. subtilis* spores have been shown to be a safe and effective vaccine carrier and adjuvant against a variety of viruses in mice [74]. Specific antigens can be expressed on the outer surfaces of spores for certain *B. subtilis* strains, such as WB800N. *B. subtilis* is not only a non-pathogenic microorganism [75]; it can also be applied as a GRAS food ingredient [76] in human foods and animal feeds. It can also tolerate the acidic environment in the digestive tract and heat [77], which enables effective delivery to the gut and enhanced stability during storage and transportation. Fajardo-Cavazos and Nicholson reported that freeze-dried *B. subtilis* spores in capsules can survive up to 3 years, not only in ambient conditions, but also in a round trip voyage to Mars with the presence of Galactic cosmic radiation and solar particle-event radiations [52]. In addition, *B. subtilis* is easy to modify genetically [78], which makes it easier to design recombinant spores targeting both the original SARS-CoV-2 and mutant viruses (Figure 1). Here, we successfully designed and engineered a type of recombinant *B. subtilis*, which can express sRBD on the surface of spores by encoding sRBD linked with the CotC gene. Our group identified the sRBD protein as an important recognition marker, suggesting that it may play an important role in stimulating antibodies to SARS-CoV-2 [79]. Consistent with other reports, the protein has been shown to bind to the host, suggesting that the sRBD protein can act as a cell-surface antigen in host–pathogen interactions [80]. The biochemical importance and biological relevance of the sRBD protein make it a promising SARS-CoV-2 vaccine antigen [81]. In our vaccination trials, the engineered *B. subtilis* showed high immunogenicity and a comparable protective effect (Figure 3 and Figure 4).

To validate the effectiveness of oral vaccines, we employed the method of the co-incubation of *B. subtilis* spores with immune cells to detect the in-vitro cytokine level. The experimental results showed that the cytokine level was greatly upregulated, proving that the *B. subtilis* spore has immunological regulation activity. In the mouse experiment, 8-week-old BALB/mice were examined with recombinant *B. subtilis* spores by oral administration. Through the detection of serum samples in each immunization regimen group, a significant increase in IgM and IgG antibodies against sRBD titer was detected. Surprisingly, a significant level of IgA antibody against sRBD was also detected in the intestinal tissue. Increased cytokine levels can also be detected through the isolation and activation of splenic cells. The observations of animal behavior and the extent of physical injury did not reveal any adverse effects, for example, changes in body weight and eating habits or any organ or tissue damage, proving that the engineered *B. subtilis* was safe for mice.

Subsequent studies in human trials have shown that *B. subtilis* spores are believed to be safe to humans, as no adverse or side effects have occurred. Through three courses of oral administration of recombinant *B. subtilis*, the levels of neutralizing antibody against sRBD were elevated, demonstrating that the *B. subtilis* could stimulate the mucous membrane in the gut to generate an immune response. The results of this study provide insights for the development of novel COVID-19 orally administered vaccines and encourage large-scale production in the future. Advances in engineering experiments with *B. subtilis* could help in applying the method to prevent other viral infections, such as influenza.

Coronavirus is a virus that invades various organs of the human body through the respiratory tract [82], and the biggest damage to the host is often caused by the sRBD spike protein on its surface [82]. Therefore, we proposed that the oral vaccine administered through the gastrointestinal tract may induce a systemic protective effect [83]. Furthermore, oral vaccines can provide convenience in practical application. In this context, to supplement the current coronavirus injection vaccine strategies, the results of this study provide an alternative route of administration for future vaccine developments.

Given the GRAS properties of *B. subtilis* [84], a preliminary human trial with a dose level derived from the no-observed-adverse-effect level (NOAEL) in the mouse study was conducted, which was equivalent to 5 × 10^7^ spores/kg/day. The dose chosen was found to be much lower compared with other human studies regarding the treatment of genetically modified gut microbiomes, such as the use of *Escherichia coli* strain SYNB1020 in a phase 1 dose-escalation study (1.5 × 10^12^ colony forming units for up to 14 days [70]). Based on the limited number of health human volunteers, our study showed no observable adverse health events after three courses of dosing of the spore of *B. subtilis* (a total of 9 days in 4 weeks). Surprisingly, the immune response of the volunteers at such a low dose level could also be significantly increased after three courses of oral dosing. The study can provide supportive information to further studies regarding the safety and efficacy in forthcoming clinical development.

The traditional design of vaccines has focused on producing whole spike protein antigens in the vaccines, while the proposed oral vaccination in this study focuses on the expression of sRBD on the spores of *B. subtilis.* Due to the similar immunological response observed, our study suggested a more specific antigen for use in generating antibodies.

Our oral vaccine is an attractive vaccine delivery system with high protective efficacy, safety, temperature stability, simplicity of preparation and low cost. Spores of *B. subtilis* are generally stable under harsh environments during storage and transportation. Persistent sRBD antigens expressed on the surface of recombinant *B. subtilis* spores can enhance the shelf life of the vaccines [85]. The good stability of oral vaccines at room temperature plays an important role in the effectiveness and distribution of vaccines. Our *B. subtilis* spores were shown to be stable for at least 6 months of storage at room temperature. This overcomes the requirement of vaccine stability at room temperature, which will be a potential advantage for future group immunity worldwide.

In addition to the potential clinical benefits of the careful selection and combination of virus epitopes, oral vaccines have several technical advantages over inactivated, attenuated, or viral vector vaccines, including the possibility of mass production in dedicated fermenters and the lower risk of contamination with residual pathogens. Another advantage of this *B. subtilis* oral vaccine platform is that the antigen could be easily amended to an upcoming variant by modifying only the DNA sequence of the plasmid.

In the context of the ongoing COVID-19 pandemic, where large and easy-to-use vaccine supplies are needed, we have provided a potential candidate for oral vaccination. The manufacturing of genetically modified bacteria is a well-developed strategy. The supply of freeze-dried *B. subtilis* spores in capsule form can maintain the shelf life of vaccines for long-term storage under ambient conditions, which has the advantage of the allocation of vaccines to some rural areas. Oral administration is expected to overcome significant technical limitations associated with vaccination, including avoiding needles as additional equipment for distribution, making those who have a fear of needles more comfortable, and the ability to self-medicate, especially in developing countries. In addition to the ease of use, the option of an oral booster vaccine may benefit patients who have had adverse reactions to previous injections.

## 5. Conclusions

In summary, a stable and effective recombinant *B. subtilis* spore displaying the sRBD of SARS-CoV-2 on the cell surface was produced. In our human pilot study, no adverse health event was observed in healthy volunteers after the administration of *B. subtilis* spores. Increases in antibodies against sRBD in unvaccinated mice and humans after oral administration were also found. The *B. subtilis* spore elicits a variety of adaptive immune responses, which are expected to be good candidates for COVID-19 oral vaccines. The results of this study warrant the further clinical development of *B. subtilis* spores as an oral vaccine candidate against COVID-19.

## 6. Patents

Patents resulting from the work reported in this manuscript were filed with Chinese (patent no. 202111143384.9), Hong Kong (patent no. 32021042343.2) and PCT patents.

## Figures and Tables

**Figure 1:** (**A**) Schematic representation of DNA constructs: a. pHT01-DT-A-sRBD; b. pHT01-DT-B-sRBD; c. pHT01-DT-C-sRBD constructed for displaying sRBD on the surface of the spore. Arrows indicate the directions of gene expression. (**B**) Schematic representation of the steps to produce the *B. subtilis* spores. (**C**) Western blot analysis of sRBD expressed by various constructs (Lane 1: sRBD standard; Lane 2: pHT01-DT-A-sRBD; Lane 3: pHT01-DT-B-sRBD; Lane 4: pHT01-DT-C-sRBD). (**D**) Western blot analysis of sRBD expressed by pHT01-DT-C-sRBD at various times after 1mM IPTG induction. All sample wells were equally loaded with same amount of cell lysates. Three independent experiments were performed with similar results.

**Figure 2:** (**A**) Immunofluorescent staining of sRBD protein on recombinant *B. subtilis* spores visualized under the fluorescent microscope. Three sRBD expression constructs linked with different coating proteins, CotA, CotB and CotC, were cloned and transformed into *B. subtilis* WB800N strain for protein expression. Only the CotC-linked sRBD protein was able to display sRBD on the surface of recombinant *B. subtilis spores.* (**B**) Flow cytometry of recombinant *B. subtilis* spores transformed with empty vector pHT-01 and CotC-linked sRBD expression construct. The CotC-linked sRBD expressed *B. subtilis* spores were immunoreactive to anti-sRBD (indicated by a red arrow).

**Figure 3:** (**A**) Dendritic cell cultures were treated with peptidoglycan from *B. subtilis* (PGN-BS, 2.5 μg/mL) or PBS for 48 h, and the cell media were collected for cytokine profiling. Proinflammatory factor (TNF-α, IL-1β, IL-6, and IL-10) concentrations from dendritic cells were measured. Number of independent experiments = 3. (**B**) Dendritic cell cultures were co-treated with PGN-BS and/or Poly(I:C) HMW for 48 h, and the cell media were collected for cytokine profiling. Proinflammatory factor (TNF-α, IL-1β, IL-6, and IL-10) concentrations from dendritic cells were measured. Number of independent experiments = 3. (**C**) Dendritic cell cultures were co-treated with recombinant spores and/or Poly(I:C) HMW for 48 h, and the cell media were collected for cytokine profiling. Proinflammatory factor (TNF-α, IL-1β, IL-6, and IL-10) concentrations from dendritic cells were measured. Data presented as mean ± SEM. Number of independent experiments = 6. * *p* < 0.05, ** *p* < 0.01, *** *p* < 0.001, one-way ANOVA with Tukey’s post hoc test.

**Figure 4:** (**A**) Schematic diagram for oral vaccine administration and serum collection. Three doses of 1 × 10^9^/kg engineered *B. Subtilis* spores expressing the sRBD of SARS-CoV-2 were administered to 8-week-old BALB/c mice orally at days 1–3, 14–16, and 28–30. The blood samples of mice were collected at days 0, 8, 22, and 38 for subsequent ELISA analysis in measuring the IgG antibody level against sRBD. (**B**) The serum IgG levels in the spike protein were quantified by ELISA. A gradual increase in IgG level was observed after the second and third doses of *B. subtilis* spores. * *p* < 0.05, *** *p* < 0.001, two-way ANOVA with Tukey’s post-hoc test.

**Figure 5:** (**A**) Schematic presentation of the immunization schedule in humans. Healthy volunteers were orally administered with 5 × 10^7^ spores/kg person of *B. subtilis* spores for three courses. (**B**) The antibody titers targeting the RBD of SARS-CoV-2 were measured with a CLIA-based assay. Each connected dot represents one individual. (**C**,**D**) Representative plot of pseudovirus neutralizing assay. Serum samples from immunized volunteers were pre-incubated with wild type (**C**) or D614G (D) SARS-CoV-2 pseudoviruses carrying a GFP reporter gene and added to human lung carcinoma cell A549 expressing human ACE2 and TMPRSS2. The percentages of infected cells over serum dilution were fitted with non-linear regression. (**E**,**F**) The serum dilution resulting in a 50% reduction in infection was designated as EC_50_. Each connected dot represents one individual. ** *p* < 0.01, *** *p* < 0.001, two-way ANOVA; number of volunteers = 6.

## Data Availability

The data that support the findings of this study are available from the corresponding author, K. Kwong, upon reasonable request.
